# *Clerodendrum wallichii* Merr Methanol Extract Protected Alcohol-Induced Liver Injury in Sprague-Dawley Rats by Modulating Antioxidant Enzymes

**DOI:** 10.1155/2022/5635048

**Published:** 2022-08-23

**Authors:** Yujian Tian, Ning Liang, Tao Jing, Fang Yuan, Md. Moklesur Rahman Sarker, Mohammad Rifat Alam Maruf, Shuai Chen

**Affiliations:** ^1^Department of General Surgery, The 904 Hospital of PLA Joint Logistic Support Force (Wuxi Taihu Hospital), Wuxi, Jiangsu 214044, China; ^2^Department of Clinical Laboratory, Haikou Health Service Center, Haikou, Hainan 570208, China; ^3^Department of Hepatobiliary Surgery, Qilu Hospital Huantai Branch, People's Hospital of Huantai County, Shandong, Huantai 256400, China; ^4^Department of Clinical Laboratory, Shanxi Jincheng People's Hospital, Jincheng, Shanxi 048000, China; ^5^Department of Pharmacy, State University of Bangladesh, 77 Satmasjid Road, Dhanmondi, Dhaka 1205, Bangladesh; ^6^Pharmacology and Toxicology Research Division, Health Med Science Research Limited, 3/1 Lalmatia, Dhaka 1207, Bangladesh; ^7^Department of General Surgery, The Affiliated Hospital of Jiaxing University, Jiaxing, Zhejiang 314001, China

## Abstract

**Materials and Methods:**

An oral acute toxicity study was carried out following OECD guidelines. Hepatotoxicity was induced by the administration of ethanol for 4 weeks. Hepatic enzymes and oxidative stress biomarkers were determined using commercial diagnostic kits.

**Results:**

Treatment of rats with MECW (800 mg/kg) showed the highest reduction of body weight (4.76 ± 0.372 vs. 16.92 ± 0.846) and liver weight (3.06 ± 0.128 vs 5.55 ± 0.311). Treatment of rats with MECW at 200, 400, 600, 800, and 1000 mg/kg significantly (^*∗∗*^*p* < 0.01) reduced SGPT. Similarly, serum SGOT and ALP were significantly decreased by MECW (200, 400, 600, 800, and 1000 mg/kg). All used doses of MECW significantly increased antioxidant enzymes GSH and SOD. MECW (600 and 800 mg/kg) significantly promoted CAT levels in liver tissues; whereas, it significantly diminished oxidative biomarker, MDA. Histopathological observations of the liver showed improvement in the architecture of hepatic cells having signs of protection with a reduced number of inflammatory cells, vascular degeneration and congestion, cellular degeneration, necrosis, and significant reduction of fatty cells accumulation. Acute toxicity study resulted in the well-tolerability and safety of used doses of MECW (200–1000 mg/kg) in rats.

**Conclusion:**

Our study clearly demonstrated the hepatoprotective effect of *Clerodendrum wallichii* extract against ethanol-induced liver injury in the laboratory rats model.

## 1. Introduction

*Medicinal plants and isolated bioactive compounds are a good hub for the discovery and development of novel therapeutics. Due to the adverse effects and toxicity issues of synthetic drugs, scientists all over the world are emphasizing natural medicines and phytocompounds for the treatment of chronic as well as emerging diseases such as diabetes* [1–7], *cancer* [8, 9]*, immunological disorders* [10–17]*, hyperlipidemia* [18, 19]*, obesity* [20]*, neurological diseases* [21–23]*, inflammation* [24, 25]*, diarrhea* [26, 27]*, infections* [28], *and renal impairment* [29]. Clerodendrum is a genus of 500 species (family Lamiaceae) and is widely distributed across the world. *Clerodendrum wallichii* Merr (family: Lamiaceae) is a tall ornamental bushy shrub with pendulous white flowers which is native to Southern Asia and Southern China, found in hilly areas [30]. In China, *Clerodendrum wallichii* is found in open forests on mountain slopes. The leaves of the plant have been used in the traditional system of medicines for the treatment of fever, skin infections, inflammation, diarrhea, and dysentery [31]. Some tribal people in Asian countries eat this plant as vegetables [32]. Phytochemical investigations on this plant were reported to contain phenolic and flavonoid compounds [32, 33]. The aerial parts of *C. wallichii* were reported to possess stigmasterol, *β*-sitosterol, clerosterol, clerodolone, and 24(S) ethyl-cholesta-5,22,25-trien-3*β*-ol [32, 34]. Powder microscopic observation of *Clerodendrum wallichii* leaves was reported to contain cubic type and square type calcium oxalate crystals [31].

Phytochemical analysis of *Clerodendrum* sp. was reported to contain cardiac glycosides, terpenoids, anthraquinones, proteins, flavonoids, saponins, tannins, lignin, phenol, and alkaloids [35]. Methanol extract from the leaves of *Clerodendrum wallichii* was reported to have analgesic, antioxidant, and cytotoxic activities [30]. The hydroalcoholic extract showed antidiarrheal activity [32]. Alcoholic extract and hydroalcoholic extract showed potential anti-inflammatory activity by reducing paw edema and inhibition of the synthesis and release of inflammatory mediators through cyclooxygenase and lipoxygenase pathways [36]. Kar et al., 2020, performed GC-MS analysis of twelve *Clerodendrum* sp. which resulted in the presence of 68 phytocompounds; among them, 29 were found to be unique [37]. The major phytocompounds found in their study include triterpenoid compounds (Taraxerol, Friendelin, Betulin), fatty acids (linoleic acid, hexadecanoic acid), squalene, stigmasterol, and arbidol [37].

Although several studies have been conducted on different *Clerodendrum species*, pharmacological and biological investigations on *Clerodendrum wallichii* are scarce. No scientific investigation has been conducted to evaluate its effect on the liver and/or its functional activities. Therefore, we aimed to assess the effect of methanol extract of the leaves of *Clerodendrum wallichii* (MECW) against ethanol-induced liver injury in the laboratory rats model.

## 2. Materials and Methods

### 2.1. Collection and Identification of the Plant

Fresh whole plants of *Clerodendrum wallichii (*Merr) were collected from the hill forest of Jiangsu province of China in June 2019. Then, the plant was then identified by a Taxonomist and a voucher of plant specimen has been preserved in the Institute of Botany, Jiangsu province, China.

### 2.2. Preparation of Extract

The extract was prepared by maceration techniques [38], a type of cold extraction process to avoid the degradation of phytoconstituent(s) in the extract. Briefly, after collecting and identification, the plants were washed, dried in an oven at 40°C, and pulverized in an electric grinder to powder. Then, 500 gm of powder was soaked in 2 L of methanol in an amber glass bottle. The container was sealed by a bottle cap and kept for a period of 14 days accompanying occasional shaking and stirring two times a day to facilitate the extraction of phytoconstituents. The whole mixture was filtered by a cotton plug followed by Whatman number 1 filter paper. The filtrate was further evaporated to dryness using a rotary evaporator at 40°C temperature with pressure. The crude methanol extract of *Clerodendrum wallichii* (MECW) was prepared as a concentrated gummy mass which was then transferred to a clean beaker and evaporated the methanol residue in the extract.

### 2.3. Chemicals and Reagents

Methanol and ethanol were purchased from Merck (Germany). Silymarin (Milk Thistle) was purchased from a local pharmacy which was used as a standard hepatoprotective drug for experimental purposes. Ketamine HCl and xylazine HCl were purchased from Sigma-Aldrich (St. Louis, MO, USA). All other analytical grade reagents were locally procured and purchased.

### 2.4. Experimental Animals

Sprague-Dawley (SD) male rats weighing between 120 and 160 g, aged 6–8 weeks old, were purchased from Shanghai Laboratory Animal Center (SLAC, Shanghai, China). The rats were housed six per plastic cage provided with wood chip bedding, maintained with a 12/12 h light-dark cycle, and allowed free access to standard rodent diet and water *ad libitum*. Environmental changes were strictly controlled, and prior to any experiment, all the animals were kept for 1 week to adjust to the new housing environment.

The ethical approval was obtained from the Ethics Committee of the 904 Hospital of PLA Joint Logistic Support Force, Jiangsu, China (Approval Number: 202100987). All the experiments were conducted according to the approved Animal Use Protocol by the Ethics Committee and in accordance with the Guidelines for Care and Use of Laboratory Animals published by the US National Institutes of Health. The Federation of European Laboratory Animal Science Associations (FELASA) guidelines and recommendations were followed to reduce the pain and stress of the experimental animals. At the end of the experiments, the rats were sacrificed with anesthesia overdose: Ketamine HCl (100 mg/kg) and xylazine (10 mg/kg) through intraperitoneal route [39].

### 2.5. Experiment Design

Forty SD male rats were randomly divided into eight groups, each group contained 5 rats:

- Group 1: nonalcoholic control group (received water only, oral route)
- Group 2: alcoholic control group (ethanol 1 ml/100 gm b.w., oral route)
- Group 3: ethanol (1 ml/100 gm b.w.) + MECW (200 mg/kg b.w.)
- Group 4: ethanol (1 ml/100 gm b.w.) + MECW (400 mg/kg b.w.)
- Group 5: ethanol (1 ml/100 gm b.w.) + MECW (600 mg/kg b.w.)
- Group 6: ethanol (1 ml/100 gm b.w.) + MECW (800 mg/kg b.w.)
- Group 7: ethanol (1 ml/100 gm b.w.) + MECW (1000 mg/kg b.w.)
- Group 8: ethanol (1 ml/100 gm b.w.) + Silymarin (25 mg/kg b.w.)

The animals were treated with different doses of methanol extract of *C. wallichii* (MECW) as mentioned above for 4 weeks along with the administration of ethanol every day. Silymarin was used as a positive control (standard hepatoprotective agent).

### 2.6. Determination of Acute Toxicity Level of MECW

An oral acute toxicity study (LD_50_ determination) of methanol extract of *C. wallichii* (MECW) was performed following the OECD (Organization for Economic Cooperation and Development) guideline by Fixed Dose Procedure (OECD protocol no. 420) as followed by Kifayatullah et al., 2015 [19], and Al-Afifi et al., 2018 [40] Briefly, SD female (nulliparous and nonpregnant) rats, aged 8 weeks, were acclimatized to laboratory conditions 7 days prior to the experiment. The rats were divided into five groups, each comprising 5 animals. Group 1 served as the untreated control (received water only), and groups 2, 3, and 4 received MECW doses of 300 mg/kg, 2000 mg/kg, and 3000 mg/kg, respectively. The rats were overnight fasted for food (not water) before dosing and fasted for food 3-4 hours after the administration of doses. The animals were observed individually during the first 30 minutes after dosing; special attention was given during the first 4 hours; then, they were observed periodically during the first 24 hours to see any toxic effects in the animals. During the entire period of observation for 14 days, the animals were observed and monitored for any changes in behavior, body weight, urination, food intake, water intake, respiration, convulsion, tremor, temperature, constipation, changes in eye and skin colors, and mortality of the animals.

### 2.7. Determination of Hepatoprotective Activity of *C. wallichii* Extract

The experimental rats were treated with different doses of *C. wallichii* extract as mentioned in the research design for 24 days. On the day 25^th^, the animals were sacrificed by anesthesia overdose followed by euthanasia [39]. The rats were observed daily for any kind of toxic effects, mortality, food intake, water, and other sorts of behavioral changes, if any. Approximately 5 mL of blood was collected from the dorsal aorta of each rat. Two milliliters of blood was dispensed into EDTA for hematological and 3 mL into heparin for biochemical analysis, respectively. The liver was excised and weighed. Liver tissue samples were stored in Bouin's fixative for histopathological observations. The remaining hepatic tissue was stored at −20°C for measurement of catalase (CAT), glutathione-S-transferase (GST), superoxide dismutase (SOD), malondialdehyde(MDA), and hydrogen peroxide (H_2_O_2_). Briefly, the frozen liver tissue samples were defrosted and homogenized in ice-cold phosphate-buffered saline. The homogenate was centrifuged at 3,000 rpm at 4°C for 10 min. Then, the supernatants were collected and assayed for the determination of CAT, GST, SOD, MDA, and H_2_O_2_ by using commercially available kits (Jiancheng, Inc., Nanjing, China) as per the procedure followed by Maimaitimin et al., 2018 [41].

### 2.8. Liver Function Test (Measurement of Liver Function Parameters)

For the evaluation of the functions of the liver in the treated and untreated rats, the levels of serum glutamic pyruvate transaminase (SGPT), serum glutamic oxaloacetic transaminase (SGOT), and alkaline phosphatase (ALP) were measured using commercial diagnostic kits (Jiancheng, Inc, Nanjing, China) as per the procedure described by Bera et al. [42].

### 2.9. Histopathological Evaluation of Liver

Histopathological experiments were performed as described by Song et al. (2018) [43]. After sacrificing the rats, livers were collected and immediately fixed in 10% buffered formalin (*pH* 7.4) and embedded in paraffin. A portion of the liver was cut (4-5 *μ*m), stained with hematoxylin-eosin (H&E), and the sections were examined with a computer-aided microscope for the determination of morphological and/or pathological changes (×600 magnification). The histological scores were assessed as mentioned by Ishak et al. (1995) [44]. The scoring systems were performed based on a sum of three parameters: inflammation grade, cell infiltration, and tissue disruption. H and *E* staining in the livers was scored using a scale of 0 to 4 (0 = no inflammation grade, cell infiltration, and tissue disruption; 1 = 0–25% inflammation grade, cell infiltration, and tissue disruption; 2 = 25–50% inflammation grade, cell infiltration, and tissue disruption; 3 = 50–75% inflammation grade, cell infiltration, and tissue disruption; and 4 = 75–100% inflammation grade, cell infiltration, and tissue disruption). Each tissue was evaluated for the sum of three parameters and by the degree of liver injury using a qualitative score that ranged from 0 to 4. A score of 0 was categorized as no damage, scores between 1 and 2 were categorized as light injury, and scores of 3 and 4 were categorized as serious injury.

### 2.10. Statistical Analysis

The data obtained from the investigation were analyzed by one-way analysis of variance (ANOVA) using Statistical Package SPSS (version 25.0) software of IBM (International Business Machines) Corporation, USA, followed by Dunnett's-T3 test to determine statistical significance between groups. The data are means ± SEM (standard error mean) of five animals. The *p* value, *p* < 0.05 was considered statistically significant.

## 3. Results

### 3.1. Effect of MECW on Body Weight and Liver Weight in Ethyl Alcohol-Treated Rats

Administration of ethanol to SD rats significantly increased both the body weight and liver weight compared to the nonalcoholic control group (Table 1). Treatment of the rats with MECW (doses 400, 600, 800, and 1000 mg/kg) and the standard hepatoprotective drug, silymarin (25 mg/kg), significantly (^*∗*^*p* < 0.05, ^*∗∗*^*p* < 0.01, ^*∗∗∗*^*p* < 0.001) reduced both the body weight and liver weights in alcoholic rats. The highest reduction of body weight and liver weight was observed by MECW at the dose of 800 mg/kg (4.76 ± 0.372 vs. 16.92 ± 0.846 for body weight and 3.06 ± 0.128 vs 5.55 ± 0.311 for liver weight) compared to the untreated alcoholic control group. This significant reduction has almost changed the body weight and liver weight to the normal value when compared with nonalcoholic control.

### 3.2. Protection of Hepatic Damage by MECW in Ethanol-Intoxicated Rats

The level of hepatic enzymes was measured to evaluate the protective effect of MECW against ethanol-induced liver damage in SD rats. Our experiment resulted in the fact that the treatment of the rats with ethanol significantly elevated the levels of important hepatic enzymes SGPT, SGOT, and ALP in serum compared to the control group (Figures 1(a)–1(c)). However, further treatment of the alcohol-pretreated rats with different doses of MECW and silymarin significantly reduced the amount of all the elevated enzymes.

As we can see in Figure 1(a), treatment of the rats with ethanol at the dose of 1 mL/100 gm b.w. significantly increased the level of SGPT (^##^*p* < 0.01) compared to the control group (89.6 IU/L vs. 40 IU/L). However, further treatment of the alcohol-induced rats with MECW at the doses of 200, 400, 600, 800, and 1000 mg/kg significantly (^*∗∗*^*p* < 0.01) reduced the level of SGPT compared to the alcoholic control group. This reduction was so potential that the level of SGPT reduced to the normal level which was observed in the serum of nonalcohol-treated rats. The highest reduction of the level of SGPT was observed by MECW at the dose of 800 mg/kg.

Similarly, the level of serum SGOT (^###^*p* < 0.001, 105.4 vs. 268 IU/L) and ALP (^#^*p* < 0.05, 126.2 vs. 359.4 IU/L) was significantly increased in alcohol-treated rats (Figures 1(b) and 1(c)). Treatment of ethanol-induced rats with MECW at the doses of 200, 400, 600, 800, and 1000 mg/kg significantly diminished the level of SGOT and ALP in comparison to only the alcohol-treated group. MECW at the dose of 600 mg/kg exhibited the highest reduction of the level of both SGOT and ALP. However, treatment with silymarin (25 mg/kg), which was used as a standard hepatoprotective agent, also significantly reduced the level of both SGOT and ALP in comparison to the alcohol control group (Figures 1(b) and 1(c)).

### 3.3. Effect of MECW on the Alcohol-Induced Oxidative Stress of Liver in Rats

For the determination of the effect of MECW on oxidative stress induced by alcohol in rats, we measured the important antioxidant liver enzymes GSH, CAT, and SOD. We have also measured MDA as an indicator of free radicals and stress in the liver. As shown in Table 2, treatment of SD rats with ethanol caused significant decreases in the level and activities of antioxidant enzymes GSH (^*∗∗∗*^*p* < 0.001; 3.18 ± 0.126 vs. 7.304 ± 0.284 *µ*g/mg protein), CAT (^*∗∗∗*^*p* < 0.001; 4.47 ± 0.234 vs. 8.73 ± 0.342 IU/mg protein), and SOD (^*∗∗∗*^*p* < 0.001; 14.57 ± 0.745 vs. 31.57 ± 1.096 U/mg protein) in the tissues of the liver when compared to the nonalcoholic control group. However, treatment of rats with all the doses of MECW significantly increased the activities and levels of GSH and SOD compared to the alcoholic control group (Table 2). MECW at doses of 600 and 800 mg/kg significantly promoted the levels of CAT in liver tissues. Silymarin at the dose of 25 mg/kg significantly enhanced the level of all the antioxidant enzymes GSH, CAT, and SOD compared to alcoholic control rats (Table 2).

On the other hand, alcohol treatment in experimental rats significantly increased the level and activity of MDA in comparison to nonalcoholic control rats (^*∗∗*^*p* < 0.001; 6.10 ± 0.335 vs. 1.81 ± 0.050). However, further treatment of the alcoholic rats with MECW significantly diminished the levels of MDA; the maximum reduction of MDA level was observed by the MECW (600 mg/kg) (^*∗∗∗*^*p* < 0.001; 1.90 ± 0.101 vs. 6.10 ± 0.335 nmol/mg protein) (Table 2).

### 3.4. Effect of MECW on Histopathological Assessment of Alcohol-Induced Liver Damage

Histopathological observation of liver sections of the nonalcoholic control group showed normal cellular architecture, distinct hepatic cells, sinusoidal spaces, central vein, and no accumulation of fat (Figure 2(a)). In the ethanol-treated group (Figure 2(b)), hepatic cells were found to have centrilobular necrosis, hyperplasia, cellular degeneration, inflammation, polymorphonuclear aggregation, and accumulation of fats. The rats treated with MECW (400, 600, 800, and 1000 mg/kg) (Figure 2(d)–2(g)) and Silymarin (25 mg/kg) (Figure 2(h)) showed almost normal architecture of the hepatic cells having the signs of protection with the reduced number/absence of inflammatory cells, vascular degeneration and congestion, cellular degeneration, necrosis, and significance reduction/absence of fatty cells accumulation.

### 3.5. Oral Acute Toxicity Study of MECW

The oral acute toxicity study of MECW was carried out following OECD guideline-Fixed Dose Procedure (OECD protocol no. 420) as mentioned in the Methodology section. No case of mortality was observed during the 14 days of treatment with a limit dose of 3000 mg/kg BW of MECW. All the treated animals could tolerate the MECW doses, and there was no statistically significant difference in body weight between the treated and untreated groups. The animals did not exhibit any abnormalities or major behavioral changes such as respiratory distress, abnormal locomotion, tremors, salivation, diarrhea, sleep, walking backward, reaction to handling, catalepsy, coma, or any toxic symptoms either immediately or during the posttreatment observational period of 14 days. Thus, we can say that the LD_50_ for oral administration of MECW is higher than 3000 mg/kg BW Therefore, the used doses of MECW (200–1000 mg/kg) were well tolerated by the animals (data not shown).

## 4. Discussion

The present study evaluated the hepatoprotective activity of methanol extract of leaves of *Clerodendrum wallichii* Merr against chronic administration of ethanol-induced liver injury in SD rats. The liver is impaired or damaged or injured by several factors such as chemicals including alcohol [45], drugs [46], viruses [47], and stress [48]. In our investigation, we used ethanol to induce hepatotoxicity as ethanol is clinically relevant. Our experiments clearly demonstrated the hepatoprotective activity of MECW by reducing the secretion of important hepatic enzymes, namely, SGPT, SGOT, and ALP in serum which were started to produce highly with the treatment of rats with ethanol (Figures 1(a)–1(c)). The highest reduction of the amount of SGPT, SGOT, and ALP was exhibited by the MECW at the doses of 800 mg/kg, 600 mg/kg, and 600 mg/kg, respectively. These doses diminished the levels of the hepatic enzymes in ethanol-induced rats to the level of normal value of the ethanol-untreated rats. This demonstrates that the MECW potentially showed hepatoprotective activity by lowering the secretion of important hepatic enzymes to restore to normal levels; this effect was even stronger than that of standard hepatoprotective agent silymarin (25 mg/kg).

ALT (previously known as SGPT) and AST (known as SGOT) are aminotransferases that catalyze the interconversion of amino acids and alpha-oxo-acids by transfer of amino groups. AST is present in the cytoplasm as well as in the mitochondria of the hepatic cells whereas ALT is present in the cytoplasm of hepatic cells [49]. Both the ALT and AST are present in hepatocytes in large amounts relative to serum. Serum AST, ALT, and ALP are useful biomarkers of liver injury. The presence of a high amount of either ALT or AST or both in blood plasma is an indicator of injury or damage to hepatic cells. In our investigation, chronic administration of ethanol to the rats caused liver injury or damage-necrosis of hepatocytes which caused the release of a high amount of AST and ALT from the cytoplasm and mitochondria of hepatocytes to the blood plasma. Further treatment of alcoholic-treated rats with different doses of MECW could completely prevent hepatic impairment or damage which is clearly understandable from the normal value of ALT and AST in the blood plasma of MECW-treated animals.

The enzyme ALP is present in the cell membranes of organs that exhibit high excretory or absorptive capacity including cells lining liver sinusoids, epithelial cells of renal tubules, brush border cells of the small intestine, salivary epithelial cells, etc. The ALP is bound to the cell membranes or microsomes [49]. ALP facilitates the transfer of metabolites such as lipids, proteins, and carbohydrates across cell membranes. The normal serum range of alkaline phosphatase is 44 to 147 IU/L [50]. The ALP test is used to detect blocked bile ducts, liver damage, or bone disorders. When liver cells are damaged, it releases increased amounts of ALP into the blood. A high level of ALP in serum indicates large bile duct obstruction or infiltrative diseases of the liver [51]. In our observation, we found that ethanol treatment to the experimental rats elevated ALP levels almost 3 times compared to nonalcoholic rats. This means chronic administration of ethanol caused hepatic impairment or injury of hepatic cells or cirrhosis or necrosis. Treatment of alcoholic rats with different doses of MECW completely prevented hepatic impairment and restored the serum level of ALP to normal as compared with the nonalcoholic untreated rats group (Figure 1(c)).

The phytochemical analysis of the methanol extract of *Clerodendrum wallichii* has not been performed in this study. Previous studies reported that *C. wallichii* contains phenolic and flavonoid compounds [32, 33]. Recently, Kopilakkal et al. [52] reported hepatoprotective activity of ethanol extract of *Clerodendrum paniculatum* flowers (another *Clerodendrum* species) against carbon tetrachloride-induced hepatotoxicity in rats [52]. They also reported that the fraction of the extract rich in flavonoid contents exhibited better hepatoprotective activities *in vitro*. GC-MS and HPTLC analysis of the flavonoids/phenolic rich fraction of the extract identified 5 major compounds that were supposed to be responsible for its hepatoprotective activity which include gallic acid, quercetin, glyceric acid, pangamic acid, and pilocarpine [52]. Quercetin is a potent antioxidant flavonoid, specifically a flavonol. Gallic acid is an antioxidant phenolic compound. Another study conducted by Zhen et al. (2017) reported the potential antioxidant and hepatoprotective ability of polyphenols and flavonoids [53]. Therefore, the possible principal phytocompounds responsible for the exhibited hepatoprotection of methanol extract of *Clerodendrum wallichii* (MECW) against liver injury by modulating antioxidant enzymes are assumed to be polyphenols and/or flavonoid compounds which may include gallic acid, quercetin, and kaempferol. However, the actual bioactive phytocompound(s) responsible for hepatoprotective action would be determined by extensive phytochemical analysis for the isolation of phytocompounds and further evaluation of isolated compounds for hepatoprotective activities which may lead to bioassay-guided hepatoprotective drug discovery.

## 5. Conclusion

Our study clearly demonstrated that MECW has a strong hepatoprotective ability against ethanol-induced liver injury in experimental rats. The hepatoprotective activity of MECW was exhibited by controlling the levels of oversecretion of hepatic enzymes and promoting the antioxidants of hepatocytes restoring them to the normal level. However, further investigations are warranted.

## 6. Limitation of the Study

In this study, we have evaluated the hepatoprotective activity of *Clerodendrum wallichii* Merr. methanol extract in an animal model. Due to lack of time, we could not isolate the bioactive phytochemicals and evaluation of the isolated compounds for their hepatoprotective activity. However, we will next study the identification and isolation of bioactive compounds responsible for the potential hepatoprotective activity and its toxicological profile as well following bioassay-guided drug discovery guidelines.

## Figures and Tables

**Figure 1:** Effects of different doses (200–1000 mg/kg) of MECW and silymarin (25 mg/kg) on oxidative stress in alcohol-induced SD rats. ALT (a); AST (b); ALP (c). ^#^^,^^##^^,^^###^ significantly differs compared to the nonalcoholic control group. ^*∗*^^,^^*∗∗*^^,^^*∗∗∗*^ significantly differs compared to the alcoholic control group. The values were reported as the means ± SEM (*n* = 5 rats/group). *P* < 0.05 were considered to be significant (one-way ANOVA followed by Dunnett T3 Post Hoc test).

**Figure 2:** Representative photomicrographs of liver histopathology. Liver sections from SD rats group of nonalcoholic control (a), alcoholic control (b), MECW 200 mg/kg (c), MECW 400 mg/kg (d), MECW 600 mg/kg (e), MECW 800 mg/kg (f), MECW 1000 mg/kg (g), and silymarin 25 mg/kg (h), respectively.

**Table 1:** Effect of methanol extract of *Clerodendrum wallichii* (MECW) on the percentage change of body and liver weights in alcohol-treated SD rats.

Treatment group	Dose	Change of body weight (%)	Change of liver weight (%)
Nonalcoholic control	None	4.46 ± 0.242	3.04 ± 0.176
Alcoholic control	(ethanol 1 mL/100 g b.w. of rats)	16.92 ± 0.846^*a*^^*∗∗*^	5.55 ± 0.311^*a*^^*∗∗*^
*C. wallichii* + ethanol	200 mg/kg	13.44 ± 0.297^*a*^^*∗∗∗*^^*b*^^*∗*^	4.57 ± 0.154^*a*^^*∗∗*^
*C. wallichii* + ethanol	400 mg/kg	12.26 ± 0.653^*a*^^*∗∗*^^*b*^^*∗∗*^	3.71 ± 0.159^*b*^^*∗*^
*C. wallichii* + ethanol	600 mg/kg	8.42 ± 0.658^*a*^^*∗*^^*b*^^*∗∗∗*^	3.15 ± 0.062^*b*^^*∗*^
*C. wallichii* + ethanol	800 mg/kg	4.76 ± 0.372^*b*^^*∗∗∗*^	3.06 ± 0.128^*b*^^*∗∗*^
*C. wallichii* + ethanol	1000 mg/kg	7.28 ± 0.365^*a*^^*∗∗*^^*b*^^*∗∗*^	3.16 ± 0.104^*b*^^*∗*^
*Silymarin* + ethanol	(25 mg/kg)	3.54 ± 0.290^*b*^^*∗∗∗*^	2.99 ± 0.095^*b*^^*∗∗*^

Values are expressed as means ± SEM of five rats in each group. ^*a*^Data differed significantly (*P* < 0.05) when compared to the nonalcoholic control group within the respective column. ^*b*^Data differed significantly (*P* < 0.05) when compared to the alcoholic control group within the respective column.

**Table 2:** Effect of methanol extract of *Clerodendrum wallichii* (MECW) on oxidative stress in ethanol-induced toxicity of SD rats.

Treatment group (*n* = 5)	GSH (*µ*g/mg protein)	CAT (IU/mg protein)	SOD (U/mg protein)	MDA (nmol/mg protein)
Nonalcoholic control	7.304 ± 0.284	8.73 ± 0.342	31.57 ± 1.096	1.81 ± 0.050
Alcoholic control (ethanol 1 mL/100 g b.w. of rats)	3.18 ± 0.126^*a*^^*∗∗∗*^	4.47 ± 0.234^*a*^^*∗∗∗*^	14.57 ± 0.745^*a*^^*∗∗∗*^	6.10 ± 0.335^*a*^^*∗∗*^
*C. wallichii* (200 mg/kg) + ethanol	4.77 ± 0.277^*b*^^*∗*^	5.59 ± 0.263	24.78 ± 0.693^*b*^^*∗∗∗*^	2.30 ± 0.208^*b*^^*∗∗*^
*C. wallichii* (400 mg/kg) + ethanol	5.78 ± 0.328^*b*^^*∗∗*^	6.42 ± 0.305	25.4 ± 0.977^*b*^^*∗∗*^	2.0 ± 0.107^*b*^^*∗∗*^
*C. wallichii* (600 mg/kg) + ethanol	6.57 ± 0.218^*b*^^*∗∗∗*^	8.10 ± 0.294^*b*^^*∗∗*^	28.38 ± 0.321^*b*^^*∗∗∗*^	1.90 ± 0.101^*b*^^*∗∗*^
*C. wallichii* (800 mg/kg) + ethanol	6.31 ± 0.129^*b*^^*∗∗∗*^	7.65 ± 0.337^*b*^^*∗*^	27.72 ± 0.380^*b*^^*∗∗∗*^	1.96 ± 0.136^*b*^^*∗∗*^
*C. wallichii* (1000 mg/kg) + ethanol	5.87 ± 0.210^*b*^^*∗∗∗*^	7.28 ± 0.402	27.36 ± 0.662^*b*^^*∗∗∗*^	2.11 ± 0.179^*b*^^*∗∗*^
*Silymarin* (25 mg/kg) + ethanol	6.30 ± 0.247^*b*^^*∗∗*^	7.8 ± 0.314^*b*^^*∗*^	27.52 ± 0.402^*b*^^*∗∗∗*^	1.92 ± 0.135^*b*^^*∗∗∗*^

Effects of different doses (200–1000 mg/kg) of MECW and silymarin (25 mg/kg) on oxidative stress in alcohol-induced SD rats. GSH: glutathione; CAT: catalase; SOD: superoxide dismutase; MDA: malondialdehyde. ^*a*^^*∗∗*^^,^^*a*^^*∗∗∗*^ significantly differs compared to the nonalcoholic control group. ^*b*^^*∗*^^,^^*b*^^*∗∗*^^,^^*b*^^*∗∗∗*^ significantly differs compared to the alcoholic control group. The values were reported as the means ± SEM (*n* = 5 rats/group). *P* < 0.05 were considered to be significant (one-way ANOVA followed by Dunnett T3 Post Hoc test).

## Data Availability

All the relevant data obtained from the study have been included in the manuscript. Further details on data can be provided by the corresponding author on request.
